# Computed Tomography Image under Three-Dimensional Reconstruction Algorithm Based in Diagnosis of Renal Tumors and Retroperitoneal Laparoscopic Partial Nephrectomy

**DOI:** 10.1155/2021/3066930

**Published:** 2021-10-06

**Authors:** Haijie Zhang, Fu Yin, Liyang Yang, Anqi Qi, Weiwei Cui, Shanshan Yang, Ge Wen

**Affiliations:** ^1^Department of Imaging, Nanfang Hospital, Southern Medical University, Guangzhou 510515, China; ^2^PET/CT Center, Department of Nuclear Medicine, The First Affiliated Hospital of Shenzhen University, Shenzhen 518000, China; ^3^School of Information Engineering, Shenzhen University, Shenzhen 518000, China

## Abstract

This study was to explore the clinical application value of computed tomography (CT) images based on a three-dimensional (3D) reconstruction algorithm for laparoscopic partial nephrectomy (LPN) in patients with renal tumors. 30 cases of renal cell carcinoma (RCC) patients admitted to the hospital were selected as the research objects and were rolled into two groups using a random table method. The patients who received PLN under the three-dimensional reconstruction and laparoscopic technique were included in the experimental group (group A), and the patients who received LPN using CT images only were included in the control group (group B). In addition, the treatment results of the two groups of patients were compared and analyzed. *Results*. The effective rate of the established model was 93.3%; the total renal arteriovenous variability of group A (13.3%) was higher than that of group B (6.7%), and the operation time (131.5 ± 32.1 minutes) was much lower than that of group B (158.7 ± 36.2 minutes), showing statistical significance (*P* < 0.05). *Conclusion*. CT images based on 3D reconstruction algorithms had high clinical application value for LPN in patients with renal tumors, which could improve the efficiency and safety of LPN.

## 1. Introduction

For early renal cell carcinoma (RCC), especially small RCC with a tumor diameter of less than 4 cm, the therapeutic effects of LPN and laparoscopic radical nephrectomy (LRN) are basically the same [1]. Because LPN only removes the tumor and part of the kidney tissue, the overall renal function after surgery is better than LRN [2]. Existing studies believe that LPN should be selected for isolated patients or patients with other diseases in the contralateral kidney. Compared with traditional open surgery, LPN not only greatly shortens the prognosis and hospitalization time of the patient but also reduces the economic burden of treatment for the patient and relieves the prognosis pain of patients due to surgery greatly [3, 4]. There are two approaches for LPN, namely, transabdominal and retroperitoneal. With the continuous updating of surgical instruments and the development of laparoscopic surgery technology in recent years, the retroperitoneal approach has gradually become a hot spot for scholars. In the past, conventional laparoscopy showed in two-dimensional (2D), which was difficult to achieve the ideal diagnosis and treatment effect. Moreover, in traditional medical imaging inspections, doctors mainly use tomographic images of a certain part of the human body and usually present the imaging results in two-dimensional images such as films or display screens. The result of this method is that the image results obtained are only judged by the personal subjective experience of the doctor. The doctor can only observe the subtleties of the image with the naked eye and the lack of objective evidence to support it, which may delay the condition of the patient [5].

With the continuous development of science and technology, medical imaging technology is also being updated simultaneously, making it possible to make up for the shortcomings in traditional imaging. In recent years, reports on three-dimensional (3D) reconstruction medical imaging technology are not uncommon, which have attracted widespread attention [6]. It uses visualization technology to provide greater assistance for the optimization of imaging effects, and the resulting images have a strong sense of reality, allowing doctors to observe and analyze images from multiple angles and levels. Studies have found that the use of the built-in software of the CT equipment can generate 3D reconstruction images, such as CT angiography (CTA) and CT urography (CTU), and obtain some reference information of the 3D anatomical structure with renal tumor and renal pedicle blood vessels (RPBV) [7]. However, this method does not use 3D image segmentation technology, so it is impossible to obtain a transparent and clear display of the organ structure image. In addition, the method does not use image fusion technology, so it cannot fuse the reconstructed model data information of multiple phases. The image information obtained is relatively scattered. Although it can provide valuable reference information for disease diagnosis, it cannot provide assistance for surgical planning, so the image obtained by this method cannot be called a true 3D reconstruction image [8].

Therefore, the study intended to explore the clinical application value of CT images based on a 3D reconstruction algorithm for LPN of patients with renal tumors by constructing a 3D reconstruction model of the kidney, so as to improve the efficiency and safety of LPN.

## 2. Materials and Methods

### 2.1. Research Objects

Thirty cases of renal cell carcinoma (RCC) patients admitted to the hospital from September 2018 to September 2019 were selected as the research objects and were rolled into two groups using a random table method. The patients who received PLN under the three-dimensional reconstruction and laparoscopic technique were included in the experimental group (group A), and the patients who received LPN using CT images only were included in the control group (group B). In addition, the treatment results of the two groups of patients were compared and analyzed. There were 15 cases in group A, including 8 males and 7 females, and they were 26∼69 years old (with an average age of 52.40 ± 11.8 years). There were 15 cases in group B, including 9 males and 6 females, and they were 24∼70 years old (with an average age of 50.5 ± 10.2 years). None of the selected patients had a previous medical history of contraindications for surgery, and none of them had any hypersensitivity to contrast agents. This study was approved by the hospital ethics committee, and all selected patients had signed the informed consent.

### 2.2. Variant Type of RPBV

Classification criteria of the renal artery were defined as follows: multiple renal arteries: there were other renal artery branches in addition to the main renal artery; premature renal artery branches: renal artery branches located at a distance ≤20 mm from the opening of the renal artery; and mixed type: a combination of above conditions.

Classification criteria of renal veins were defined as follows: multiple renal veins: the main branches of the renal veins could not merge into one branch before entering the kidney but still presented as branches; abnormal renal veins: the left renal vein run behind the left renal artery, the right renal artery run in front of the inferior vena cava, and there were 2 inferior vena cava; renal veins are abnormal: renal veins were anastomosed with reproductive veins and lumbar veins, respectively; others: renal tumor compressed the renal veins, causing deformation, and so on.

### 2.3. CT Scanning

A 64-slice spiral CT (Philips, Brilliance 64, Netherlands) was used for CT scanning. Before the scan, the patient was required to fast for 3 hours and drink 500 mL of water to fill the gastrointestinal tract, so as to enhance the contrast with the kidney tissue. In addition, the breathing exercises of patients had to be trained to minimize the artifacts caused by the breathing exercises on the CT scan, so as to ensure the reliability of collected data. The standard parameters of kidney CT scan were set to the following: the tube voltage was 120 kv, the tube current was 300 mA, the time per rotation was 0.5 s, the pitch was 0.984, the layer thickness was 5 mm, and the time for the tube to rotate a cycle was 0.5 s.

At the beginning of the scan, the patient was required to maintain a supine position and performed with CT plain scan and enhanced scan sequentially from the cartilage at the xiphoid process to the plane of the pubic symphysis. During the scanning, the patient was instructed to exhale and hold to the fullest body. When the contrast agent was not injected, a plain scan was performed. Then, the MEDRAD double-barreled high-pressure syringe (US) was adopted to inject the contrast agent (iopamidol solvent 370 in high concentration) intravenously at an injection rate of 5 mL/s, and the injection dose was 1.5 mL/Kg. After all the contrast agent was injected, the injection tube was flushed with a proper amount of saline, and the enhanced scan was started. The arterial phase scan setting was set as follows: the trigger threshold was set to 200 Hu, the contrast agent was injected, and the scan was performed by taking the abdominal aorta section as the region of interest (ROI). The scan in the venous phase was started from the intravenous injection of contrast agent until the delay 65 s. The scan in the excretory phase was started from the intravenous injection of contrast agent until the delay 600 s. After the scans in the above four phases were all completed, the original image with a thickness of 5 mm was thinned, and then all image data was imported into the MxView workstation equipped for the CT. Finally, all image data were recorded to a DVD disc.

### 2.4. Construction of 3D Reconstruction Model of Kidney

The key step of 3D reconstruction was image segmentation using RGM. The characteristic of RGM was to gather similar pixels to form a ROI. The specific operation method was given as follows: the data obtained from the arterial phase and venous phase scans were entered into mimics 17.0 (Materialise, Belgium), and the upper and lower threshold range was set to 210–1,615 Hu. The renal tumor, renal artery, and renal vein tissue structure were segmented with the RGM, and the other renal artery and renal vein branches outside the ROI were eliminated with artificial auxiliary software. Finally, an ideal 3D reconstruction model of the kidney was constructed. The flowchart of 3D reconstruction of medical images is in Figure 1.

After X-ray passed through the substance, the relationship between output intensity and input intensity was expressed as the following equation:

(1) $$\begin{array}{c} I_{b}=I_{a}e^{-\mu △d}, \end{array}$$

where Δd referred to the propagation distance of X-ray and *μ* was the X-ray attenuation coefficient of the substance. *I*_*b*_ referred to the output intensity, *I*_*a*_ represented the input intensity, and *e* referred to the input parameter.

When the X-ray passed through different tissue structures of the human body, the relationship between output intensity and input intensity was given as follows:

(2) $$\begin{array}{c} I_{b}=I_{a}\left(e^{-\mu_{1}△d_{1}}e^{-\mu_{2}△d_{2}}e^{-\mu_{3}△d_{3}}\ldots \right). \end{array}$$

The above equation could be converted into integral form as follows:

(3) $$\begin{array}{c} I_{b}=I_{a}e^{-\int \mu \text{d}x}, \end{array}$$

where *x* refers to the propagation distance.

CT was developed on the basis of Wratten transformation, the equation of which was as below.

It was known that the integral of a certain function $\left(x,y\right)=\hat{f}\left(r,\theta \right)$ along the straight line *Z* was as follows:

(4) $$\begin{array}{c} p=\int_{-\infty }^{+\infty }f\left(x,y\right)\text{d}z\\ =\int_{-\infty }^{+\infty }\hat{f}\left(r,\theta \right)\text{d}z,\\ =\int_{-\infty }^{+\infty }\hat{f}\left(\sqrt{\sqrt{l^{2}+z^{2}}},\emptyset +\;\tan^{-1}\frac{z}{l}\right)\text{d}z. \end{array}$$

Then, the Wratten equation could be inversely transformed into $\hat{f}\left(r,\theta \right)=1/2\pi^{2}\int_{0}^{\pi }\int_{-\infty }^{+\infty }\left(1/r\;\cos\left(\theta -\emptyset \right)-l\right)\left(\partial p/\partial l\right)\text{d}l\text{d}\emptyset$.

The pixel color values of the image were collected from back to front and from front to back, and the synthesis algorithm of which from back to front was given as follows:

(5) $$\begin{array}{c} C_{b}=C_{a}\left(1-\alpha_{i}\right)+C_{i}\alpha_{i},\\ \alpha_{b}=\alpha_{a}\left(1-\alpha_{i}\right)+\alpha_{i}, \end{array}$$

where *C*_*a*_ represents the initial color, *C*_*b*_ represents the final color, and *α*_*i*_ refers to the opacity.

The synthesis algorithm from front to back was given as follows:

(6) $$\begin{array}{c} C_{b}\alpha_{b}=C_{a}\alpha_{a}+C_{i}\alpha_{i}\left(1-\alpha_{a}\right),\\ \alpha_{b}=\alpha_{i}\left(1-\alpha_{a}\right)+\alpha_{a}. \end{array}$$

During the image synthesis, *α* could continue to increase, the threshold was 1, and the transparency of the image was close to zero at this moment.

### 2.5. Evaluation of the Image Quality of 3D Reconstruction Model of the Kidney

The quality of the 3D reconstruction image was evaluated by a senior urologist and a senior imaging physician. Before the evaluation, the 3D reconstruction CT image quality scoring standard was developed according to the renal artery scoring standard of Sahani et al. [9], which was to record the branches of renal arteries and renal veins in detail. The evaluation had to be carried out in strict accordance with this standard. If the scores of individual images were different, the final score can be determined by researching relevant information and discussion of the two physicians. The specific criteria were given as follows: 1 point meant that the main renal artery (renal vein) and its first-level branches showed blurred blood vessel edges, with or without respiratory movement artifacts; 2 points meant that the main renal artery and its first- or second-level branches could be visible clearly, with smooth blood vessel edges and without respiratory movement artifacts, and the secondary branches were less than 4; 3 points meant that the main renal artery and its first, secondary, and tertiary branches were visible clearly, with smooth blood vessel edges, without respiratory movement artifacts, and the tertiary branches were less than 5; 4 points represented that the main renal artery and its first, secondary, and tertiary branches could be seen clearly, with smooth blood vessel edges, without respiratory motion artifacts, and the tertiary branches were greater than or equal to 5; and 5 points represented that the main trunk of the renal artery and its first, secondary, tertiary, and forth branches could be showed clearly, with smooth blood vessel edges and no artifacts of respiratory movement.

In this study, the standard for 3D reconstruction CT image of the kidney was set as follows: the renal vein score was greater than or equal to 4 points, which meant that 3 to 4 renal arteries could be distinguished from the reconstructed image; the renal vein score was greater than or equal to 2 points, which meant that 1∼2 renal veins could be identified based on the reconstructed image.

### 2.6. Preparation before LPN

LPN was performed using the 2D laparoscopic equipment (KARL STORZ, Germany). First, the 3D reconstruction model of renal tumor prepared above was incorporated into mimics 17.0 software, the simulated surgery function of which was adopted to observe the operation of the model in all directions, realize the surgical demonstrations, and formulate scientific and effective surgical plans. During the surgery, the surgeon was in charge of the model magnification and rotation, and the assistant took the specific operations. During this period, the image of the renal cortex was reconstructed by moderately transparent processing so that the surgeon can clearly observe the structure of the RPBV and assist in the completion of the operation.

### 2.7. Application of 3D Reconstruction Model of Kidney in LRN

The practical application of the 3D model in LRN was to guide the operation through the artificial image fusion method; that is, the 3D reconstruction model image was fused and superimposed on the 2D laparoscopic image, and the fused image was displayed on a separate screen. Based on the results of the image fusion, the LRN was performed synchronously. The whole process was led by the surgeon and the surgical assistant performed the actual operation. Renal artery and renal vein can be clearly distinguished due to the different intensity of vascular pulsation, and operations such as ligation and disconnection were adopted accordingly. In group A, the 3D reconstruction model and artificial fusion image method were applied for preoperative guidance and intraoperative RPBV positioning and ligation. After the blood vessel and ureter were separated and cut, the patient's kidneys were freed and the kidney lesions were carefully removed, and then a drainage tube was placed between the peritoneum of the posterior abdominal wall and the intra-abdominal fascia. In group B, the CTA combined with CTU images were applied to guide the operation and to locate and ligate the renal artery and renal vein. After the blood vessel and ureter were separated and cut, the patient's kidney was freed and the renal lesion tissue was carefully removed. A drainage tube was placed between the peritoneum and the intra-abdominal fascia on the posterior wall of the abdomen. All patients underwent the surgery successfully without any accidental interruption.

### 2.8. Statistical Methods

The data were processed with SPSS 20.0 software for statistical analysis. The measurement data were indicated as mean ± standard deviation ($\bar{x}$ ± *s*), and an independent sample *t*-test was used; the count data was displayed as a percentage (%), and the X2 test was used for analysis. All data were considered statistically significant with *P* < 0.05, and there was no statistical difference when *P* > 0.05.

## 3. Results

### 3.1. Basic Information

There were 8 males and 7 females in group A, with an average age of 52.40 ± 11.8 years; there were 9 males and 6 females in group B with an average age of 50.5 ± 10.2 years old. As illustrated in Figure 2, there was no obvious difference between the two groups of patients in indicators such as age, gender, tumor distribution, body mass index (BMI), tumor maximum diameter (TMD), hemoglobin value, and the number of adrenal artery branches (*P* > 0.05). All selected patients did not withdraw due to accident event.

### 3.2. Visualization Results of the 3D Reconstruction Model of the Kidney

A 3D reconstruction model of the kidney of 15 patients in group A was successfully constructed. This model can clearly show the main renal artery and its fourth-level branches and the main renal vein and its second-level branches. The renal can be visually observed through this model. The outline of the tumor more objectively and effectively reflects the size of the renal tumor and its spatial distribution with other tissue structures; the kidney collecting system showed a clear structure and natural connections; the entire kidney system structure was clearly displayed with anatomical details.  Figure 3 shows the images of image of renal tumor based on 2D CT and 3D reconstruction model for better comparison.

The use of a 3D reconstruction model of the kidney can clearly reflect the anatomical characteristics of RPBV. In Figure 4, the characteristics of renal artery variation were observed from the ventral and dorsal sides, so that the variation of the renal artery could be intuitively understood.

### 3.3. Image Quality Results of the 3D Reconstruction Model of the Kidney

Of the 15 kidney 3D reconstruction models prepared in this study, 14 cases met the standard, and the effective rate of the built model was 93.3% (as Figure 5). One case was unqualified because the patient's kidney was not filled with contrast medium enough, which resulted in fewer main branches of the renal artery in the 3D reconstruction model and incomplete display of the renal calyces in the renal collection system. Although the 3D reconstruction model of the kidney in this case was incomplete, it could still show the anatomical details of the renal artery and renal vein, so it had no effect on the LPN.

### 3.4. Classification on Variety of RPBV

Figures 6 and 7 show the comparisons on variations of renal artery vascular and variations on renal vein vascular in two groups, respectively. Most of the cases in both groups suffered from mixed renal artery variation, with 6 cases in group A and 7 cases in group B. The type of renal vein variation in group A was abnormal renal vein progression and other types, and there were only multiple vessels type renal vein variation in group B. There was no remarkable difference between the two groups in the total renal artery variation rate and renal vein total variation rate (*P* > 0.05).

### 3.5. LPN Results

All the enrolled patients were diagnosed as RCC before surgery, followed by LPN, and there were no serious complications such as conversion to open surgery and major bleeding that occurred during the surgery. The 3D reconstruction model of the kidney used in group A could objectively and truly reflect the structural characteristics of the kidney, the type of RPBV variation, and the spatial position relationship of kidney tumors. The constructed 3D reconstruction model was adopted for preoperative scientific planning, and it was fused and superimposed with the 2D laparoscopic images during the surgery. The surgery of the patients in group A was successful. As shown in Figure 8, the RPBV variant type was that the left renal vein run behind the left renal artery. The 3D model showed that it was safer and more effective to ligate and cut the renal artery running forward.

The scan data obtained from CTA combined with CTU images were applied in group B for preoperative planning. The patients in group B had successful surgeries.

### 3.6. Analysis on Efficacy

The operation time, estimated blood loss, intraoperative blood transfusion number/rate, incidence of complication, postoperative hemoglobin value, tumor recurrence number/rate, and other index values were analyzed for the two groups of patients. The results given in Figure 9 revealed that the operation time of group A was visibly lower than that of group B, and the difference was great in statistics (*P* < 0.05), while the differences in other indicators were not extreme (*P* > 0.05). In addition, there was no tumor recurrence in the two groups.

## 4. Discussion

The clinical application value of CT images based on the 3D reconstruction algorithm for LPN in patients with renal tumors was discussed in this study, so as to improve the efficiency and safety of LPN. A 3D reconstruction model of the kidney was constructed, the image quality was evaluated, and the RPBV mutation of the patient was classified according to the kidney mutation classification standard. Then, the 3D reconstruction model of the kidney was applied to LPN, and the curative effect of two groups of patients was analyzed and compared. The results revealed that the constructed 3D reconstruction model of the kidney could objectively and truly reflect the structural characteristics of the kidney, the variant type of RPBV, and the spatial position relationship of the renal tumors, which was helpful for the rational planning and design of LPN before surgery. Applying the 3D reconstruction model of the kidney in LPN could greatly shorten the operation time without complications. Such a result was basically consistent with the research results of other scholars.

Malignant renal tumors mostly occur in the renal parenchyma, accounting for more than 80%, including RCC, renal sarcoma, renal metastases, Wilms tumor, and transitional cell carcinoma that occurs in the renal pelvis and calyx [10]. The adult renal tumor has the highest incidence rate of RCC, followed by transitional cell carcinoma originating from the collecting system of the kidney, so the renal tumor is also known as RCC. The human body is most likely to develop RCC when it is over 50 years old [11]. Compared with the transperitoneal approach, the surgeon can reach the kidney faster through the retroperitoneal laparoscopic approach and hardly interfere with other organs in the abdominal cavity. In addition, the renal arteries are mostly behind the renal veins, and the retroperitoneal approach facilitates direct exposure and treatment of the renal arteries [12]. However, because the target kidney is tightly connected with adjacent organs in the operation of the retroperitoneal approach, the operation space is narrow, and improper operation may cause damage to other organs of the patient. How to locate RPBV quickly and accurately and deal with it effectively has become a difficult topic for many scholars, and a comprehensive and accurate understanding of the anatomical characteristics of RPBV before surgery has become the key [13].

Huang et al. [14] used the 3D reconstruction model of the kidney to successfully implement the “zero ischemia partial nephrectomy,” which not only effectively reduced the ischemic damage to the normal kidney during the operation but also promoted the research and development of partial nephrectomy with superselective renal artery occlusion. Xia et al. [15] reconstructed a digital 3D model of the kidney with clear blood vessel structure and strong stereo perception based on the CT scan data of preoperative patients and formulated a more reasonable surgical plan with the aid of simulated surgery; it was found that the actual operation was highly consistent with the 3D reconstruction; and based on this 3D model, clinical living kidney transplantation was successfully implemented, the prognosis was good, and there were no obvious surgical complications.

## 5. Conclusion

The conclusions of this study were summarized as follows: CT images based on the 3D reconstruction algorithm had high clinical application value for LPN in patients with renal tumors and could improve the efficiency and safety of LPN. It was necessary to further promote the application. However, there were still many shortcomings of this study. For example, the number of study subjects was small due to time and conditions, and the data results obtained had to be further researched. In future research, the number of samples had to be expanded to increase the persuasiveness of the data, so as to provide reliable reference information for clinical applications. The results of this study provided a reliable research basis for the clinical application of 3D technology and further demonstrated the good development prospects of 3D reconstruction technology in the medical field.

## Figures and Tables

**Figure 1:** The flowchart of 3D reconstruction of medical images.

**Figure 2:** Basic information of patients in two groups.

**Figure 3:** Images of renal tumor (male patient aged 48 years; the tumor was in the right kidney with the size of 4.7 cm). (a) 2D CT image of renal tumor. (b) CT image of renal tumor based on the 3D reconstruction algorithm.

**Figure 4:** 3D reconstruction model image of the renal artery. Variation type was premature renal artery branch A and B referred to the ventral renal artery and dorsal renal artery, respectively.

**Figure 5:** Image quality of the 3D reconstruction model of the kidney. (a) Abscissa showed the quality evaluation score of renal artery image; (b) abscissa showed the quality evaluation score of renal vein image.

**Figure 6:** Variations of renal artery vascular in the two groups.

**Figure 7:** Variations on renal vein vascular in the two groups. “Other” refers to the deformation and variation of the renal vein on the affected side of the kidney due to compression by a larger tumor.

**Figure 8:** Images of RPBV laparoscopy and 3D reconstruction model of the kidney.

**Figure 9:** Comparison of the curative effect of patients in the two groups. ∗ indicates that group A is observably different from group B (*P* < 0.05); OT represents the operation time, EBL represents the estimated blood loss, COIBT represents the case of intraoperative blood transfusions, IOC represents the incidence of complication, and PHL represents postoperative hemoglobin value.

## Data Availability

The data used to support the findings of this study are available from the corresponding author upon request.
